The article "Present and Future Perspective on PLK1 Inhibition in Cancer Treatment" was published in 2022. Journal: Front Oncol.

# Present and Future Perspective on PLK1 Inhibition in Cancer Treatment

**DOI:** 10.3389/fonc.2022.903016

**Published:** 2022-06-02

**Authors:** Michela Chiappa, Serena Petrella, Giovanna Damia, Massimo Broggini, Federica Guffanti, Francesca Ricci

**Affiliations:** ^1^ Laboratory of Experimental Oncology, Department of Oncology, Istituto di Ricerche Farmacologiche Mario Negri-IRCCS, Milan, Italy; ^2^ Laboratory of Molecular Pharmacology, Department of Oncology, Istituto di Ricerche Farmacologiche Mario Negri-IRCCS, Milan, Italy

**Keywords:** cell cycle, G2/M checkpoint, DNA damage response, EMT, PLK1 inhibitors, drug combination, immune response

## Abstract

Polo-like kinase 1 (PLK1) is the principle member of the well conserved serine/threonine kinase family. PLK1 has a key role in the progression of mitosis and recent evidence suggest its important involvement in regulating the G2/M checkpoint, in DNA damage and replication stress response, and in cell death pathways. PLK1 expression is tightly spatially and temporally regulated to ensure its nuclear activation at the late S-phase, until the peak of expression at the G2/M-phase. Recently, new roles of PLK1 have been reported in literature on its implication in the regulation of inflammation and immunological responses. All these biological processes are altered in tumors and, considering that PLK1 is often found overexpressed in several tumor types, its targeting has emerged as a promising anti-cancer therapeutic strategy. In this review, we will summarize the evidence suggesting the role of PLK1 in response to DNA damage, including DNA repair, cell cycle progression, epithelial to mesenchymal transition, cell death pathways and cancer-related immunity. An update of PLK1 inhibitors currently investigated in preclinical and clinical studies, in monotherapy and in combination with existing chemotherapeutic drugs and targeted therapies will be discussed.

## Introduction

Human Polo-like kinases (PLKs) are a family of serine/threonine protein kinases comprising five members: PLK1, PLK2, PLK3, PLK4 and PLK5, with PLK1 is the most studied one. PLK1 has numerous different functions, the best known ones being its key role in mitotic entry, in centrosome regulation, in coordinating the spindle assembly, in segregation of the chromosomes and in cytokinesis (1). Other functions of the protein beyond the cell cycle have also been described based on emerging new substrates found phosphorylated by PLK1.

PLK1 dysregulation has been reported in different tumor types, contributing to tumor development and progression. PLK1 is reported to be overexpressed (at both mRNA and protein level) in many tumors compared to the normal tissue counterpart, and its overexpression has been associated with poor patient outcome (2). In addition, its overexpression has in some cases been associated with resistance to therapy and its inhibition to re-sensitization to chemo- and radio-therapy (3–5).

This review discusses the recently discovered functions of PLK1, mainly in relation to DNA damage response, EMT (epithelial to mesenchymal transition), cell death (apoptosis/autophagy) and immune system, and looks at the preclinical activity of PLK1 inhibitors, both as single agents and in combination, as well as their clinical development.

## Structure and Regulation of PLK1

Very recent well written reviews have been published on PLK1 structure, regulation and its role in cancer development and therapy (6–9), and here we summarize some key features of the PLK1 protein that could help clarifying the rationale for the design of PLK1 inhibitors and their potential side effects.

PLK1 is a very highly conserved polo-like protein whose activity is a requisite for mitotic entry. PLK1 phosphorylates Cdc25C, WEE1 and MYT1 to promote activation of the CyclinB1/CDK1 complex in triggering prophase and, later on, in G2 and mitosis (10–13). PLK1 is involved in maturation of the centrosome, kinetochore formation, condensation of the chromosome, spindle assembly and cytokinesis (14). PLK1 maximum kinase activity is in the mitotic phase of the cell cycle and its expression is regulated by different phosphorylation events (15, 16).

The PLK1 protein (603 amino acids) comprises two polo-box domains (PBDs) at the C-terminal and a kinase domain (KD) at the N-terminal portion of the protein (**Figure 1**). The PBD determines the specific cellular localization where PLK1 can interact with phospho-epitopes on target substrates. Different PLK1 interacting proteins are implicated in multiple cellular processes (16). Mutations in its PBD interfere with PLK1 localization and function (17). PBD not only drives PLK1 substrate recognition and protein localization, but also abrogates the inhibitory interaction between KD and PBD, so the T-loop region of PLK1 (encompassing Thr210) becomes phosphorylated (Ser137 and Thr210) by upstream kinases (the most important being Aurora A and its co-factor Bora), achieving protein full activation (18). Interestingly, PLK1 can phosphorylate substrates already phosphorylated by itself (self-priming) or by other up-stream kinases (non self-priming); for example, the scaffold centrosome PBIP1 protein is first phosphorylated by PLK1 at Thr78, thus favouring in such a way the interaction of the PBD of PLK1 with PBIP1 and the correct localization of PLK1 to kinetochores (19). An example of non-self-priming is the WEE1 protein, which is first phosphorylated by a cyclin-dependent kinase (CDK) leading the binding motif for PBD of PLK1; in mitosis, when PLK1 levels rise, PLK1 binds to WEE1 at the PBD docking site and phosphorylates it, leading to its degradation (20). The initial phosphorylation of PLK1 by Aurora kinase A and its co-factor Bora in its kinase domain takes place in the cytoplasm and also leads to the exposure of a nuclear localization signal that allows PLK1 to be translocated into the nucleus (21). The phosphorylation status of PLK1 is not only important for its kinase activity and interaction with other proteins, but also for ubiquitination representing an important post-translation modification, affecting PLK1’s timely localization and degradation to allow correct cell cycle progression (22).

**Figure 1:** PLK1 protein domains. PLK1 structure includes two functional polo-box domains (PBDs) at C-terminal and the kinase domain at N-terminal.

Very recent data also suggest transient dimerization of PLK1 as a new mechanism underlying the activation of cytoplasmic PLK1 during G2 phase (23). These data suggest that in early G2 phase Bora facilitates PLK1 dimerization, acting as an allosteric modulator of the PLK1, that shifts from dimeric to monomeric active state; in late G2, PLK1 Thr210 phosphorylation by Aurora kinase A triggers dimer dissociation and the PLK1 monomers generated foster mitotic entry. These data are important as they may suggest the design of new allosteric compounds to mimic the Bora-PLK1 interaction, stabilizing and/or preventing the dimeric inactive conformation, hence inhibiting PLK1 activity.

## PLK1 and its Role in Genomic Stability

PLK1 is a well conserved master regulator of cell division in eukaryotic cells, particularly involved in mitosis, where its functions are well understood (21, 24); less known is its function during the interphase and its role as modulator of the DNA damage response (DDR) and checkpoint resolution after DNA damage.

The DDR comprises a complex network of proteins that sense specific types of DNA lesions and respond to them by activating the necessary DNA repair mechanisms, and timely regulating cell cycle progression through checkpoint activation, with the final aim of repairing the damage, or if the damage is too extensive to induce cell death (25, 26). It is hardly surprising, that proteins like PLK1 involved in the surveillance mechanisms of cell cycle progression are also involved in the DDR, due to the close interactions among these mechanisms. Both DDR and cell cycle regulation have the ultimate aim of preventing genomic instability and the transmission of altered DNA to daughter cells. In the last few years mounting evidence has suggested PLK1 is involved in the DNA damage checkpoints and in DNA repair mechanisms activated during the interphase, when nuclear PLK1 levels start to rise (during S-phase), and mitosis, when PLK1 reaches its peak of expression (15). During S/G2 and M phases PLK1 interacts with and regulates by phosphorylation several key factors involved in these pathways (27).

### PLK1 and Cell Cycle Progression

DNA is replicated during S-phase of the cell cycle, and faithful duplication of the genome is critical for the maintenance of genomic stability. Pre-replication complexes, assembled during G1 phase at the replication origins along the genome are remodeled in active replication forks (RFs) and closely regulated by Cdc7 and various S-phase CDKs (28). Subsequently, mini-chromosome maintenance (MCM) helicase complexes are recruited at the active RFs to unwind DNA into two single filaments (ssDNA), where RPA proteins can bind and stabilize them. This leaves the RF ready to load replicative DNA polymerases and proliferating cell nuclear antigen (PCNA) proteins to initiate DNA replication (28). PLK1 expression does not increase during replication until DNA synthesis is completed, but it has been recently demonstrated that PLK1 function is also needed during S-phase, though at low level (29, 30). Once replication starts, CDK2 activity promotes DNA replication, CDK1 and PLK1 activities (31, 32). At the same time, DNA replication restricts CDK1 and PLK1 activities, causing a contrasting feed-forward loop to prevent mitosis starting until DNA replication is completed, and to promote PLK1 activation immediately after S-phase, thus favoring a smooth progression from DNA replication to mitosis (30). Moreover, in the G1 and S phases PLK1 phosphorylates and regulates different factors involved in the formation of the pre-replicative complexes at DNA replication origins. These targets include Orc2, a component of the origin recognition complex (ORC) (33), MCM2-7, parts of the MCM complex (34), DBF4, which couples with Cdc7 to selectively phosphorylate MCM2 subunit for its release from DNA once replication is completed (34).

The importance of PLK1 regulation during DNA replication is proved by the fact that PLK1 inhibition is associated with impaired replication and slowing of S-phase progression *in vitro*, and that PLK1 phosphorylates Orc2 under replication stress to maintain replication and promote genomic stability (33). Recently, PLK1 was shown in an *in vitro* system to be essential in regulating the spatio-temporal replication program by interacting with several origin firing factors (i.e. RIF1, TRESLIN; TopBP1), and the immuno-depletion of PLK1 reduced the number of replication forks and origins firing (35), giving additional proof of the PLK1’s role also in S-phase.

In normal conditions, mitotic entry depends on the activation and accumulation of cyclin B1/CDK1 complex, otherwise kept inactive through the inhibitory phosphorylation of CDK1 at Thr14 and Tyr15 by the kinase WEE1 and membrane-associated tyrosine-and threonine-specific Cdc2-inhibitory kinase (MYT1) kinase. Cyclin B1/CDK1 complex is activated when Cdc25C phosphatase overcomes the inhibitory effect of WEE1/MYT1. In fact, once activated, CDK1 triggers a positive feedback loop by phosphorylating both Cdc25C and WEE1/MYT1 (14, 36, 37). PLK1 takes part in this positive feedback loop, promoting CDK1 activation and mitotic entry by upregulating CDK1, promoting activation of Cdc25C and inhibition of both MYT1 and WEE1, and by degradation through E3 ubiquitin ligase SCF βTrCP (20, 38, 39). PLK1 activation is boosted by Aurora kinase A which in cooperation with Bora, mediates its phosphorylation on Thr210 (18, 40). In parallel, cyclin-B1/CDK1 complex targets Bora to promote its interaction with Aurora kinase A, fostering PLK1 activation (41).

### PLK1, DDR and the Replication Stress Response

Upon DNA damage, checkpoints are activated and cell cycle progression is halted. DNA double strand breaks (DSBs) or stalled replication forks (RFs) cause local alteration of the chromatin structure, recruitment of sensors like the Mre11-Rad50-Nbs1 (MRN) complex at the damaged site and activation of two main checkpoint pathways: ATR/CHK1 and ATM/CHK2 (42). ATM/ATR are two phosphoinositide 3-kinase (PI3K)-related protein kinases that activate CHK1/CHK2 which phosphorylate inactivating Cdc25C, preventing the de-phosphorylation and activation of nuclear CDK1 and blocking cells in the G2/M phase (43). Cell cycle arrest allows time for DNA repair and rescue of stalled RFs. Local activation of ATM at the DSB site recruits DSB repair factors like 53BP1, BRCA1 and activation of CHK2, and lack of entry in mitosis (44, 45). 53BP1 facilitates DNA repair by the error-prone non-homologous end joining (NHEJ) pathway, while BRCA1 is important for the error-free homologous recombination (HR) pathway during the S/G2-phases (46).

PLK1 is one of the numerous kinases downstream effectors of the ATM and ATR cascades (47, 48). In normal conditions, PLK1 is inhibited after DNA damage recognition through two mechanisms. The first involves Bora ubiquitination, induced by direct phosphorylation of ATM/ATR on Thr501, leading to p-Bora and degradation by E3 ubiquitin ligase SCF-β-TRCP (49); the second mechanism involves the ubiquitination of several mitotic factors, including PLK1, by the anaphase-promoting complex/cyclosome (APC/C), an E3 ubiquitin ligase (50).

Recently, a complex interplay has been described between PLK1 and the HR repair. Zou and colleagues described an interaction between BRCA1 and PLK1, showing that during the activation of the DDR, BRCA1 promptly down-regulates PLK1 kinase activity, affecting its dynamic interactions with Aurora kinase A and Bora; in *BRCA1*-depleted cells PLK1 activity was higher than in control-siRNA treated cells (51). However, it remains to be defined how BRCA1 binding to Aurora kinase A-Bora-PLK1 inhibits PLK1 activity. The involvement of phosphatases, such as myosin phosphatase targeting subunit 1 (MYPT1), and/or ubiquitin-mediated proteolysis, have been put forward (50, 52). Mono-methylation of PLK1 on Lys209 by methyltransferase G9 inactivates PLK1 by antagonizing Aurora kinase A-Bora’s activation through phosphorylation at Thr210 (53); an increasing amount of methylated PLK1 in cells exposed to genotoxic agents has indeed been reported. PLK1 methylation is necessary for DNA replication and for the timely removal of DSB repair DNA binding proteins, like RPA2 and RAD51, or BRCA2 before cell cycle progression (47, 54).

PLK1 can actively regulate several proteins essential for DNA DSB repair *via* HR. For instance, PLK1 phosphorylates RAD51 on Ser14 during S/G2-phase and in response to DNA damage (55). A transient increase of p-Ser14 was seen 20–40 min after DNA damage and allowed subsequent RAD51 phosphorylation at Thr13 by casein kinase 2. This double phosphorylation of RAD51 favors direct binding to the Nijmegen breakage syndrome (Nbs1) protein, part of the MRN complex involved in the early phase of the DDR (55). PLK1 inhibition before DNA damage has been associated with increased sensitivity to ionizing radiation and reduction of BRCA1 foci formation, suggesting PLK1 as a possible regulator of HR activation (56). This hypothesis has been recently further supported, since PARP1 and CHK1 seem to be responsible for PLK1 modification to promote HR (57). Peng et al. first observed *in vitro* a timely coordinated activity of PARP1 a few seconds after DSB induction, triggering PARylation of PLK1. As a consequence, PLK1 is protected from degradation. After 10 min, PARG had removed PAR chains from PLK1, allowing CHK1 to activate PLK1 by phosphorylating residues Ser137 and Thr210, and promoting PLK1–mediated phosphorylation on Ser14 of RAD51 (57). Interestingly, the primed p-Ser14 RAD51 allowed its subsequent phosphorylation at Thr309 directly by CHK1 (57). These phosphorylation events fully activate RAD51 and promote HR repair. Using an innovative technique of RF proteome analysis to clarify the composition of RF challenged by DSB, Nakamura et al. described a new signaling pathway that illustrates the mechanism underlying HR-dependent recovery of the stalled RF after TOP1 inhibitor-induced damage (58). In their model, there was an ATM-dependent recruitment of PLK1 at the broken fork and PLK1-dependent limitation of NHEJ in mitosis, induced by phosphorylation of 53BP1 (59) and XRCC4 (60), that prevent error-prone NHEJ, and support CtIP-mediated HR (58). After prolonged replication stress in S phase, PLK1 has been reported to interact with 53BP1 and BRCA1, which counteract each other to protect stalled RFs and promote replication restart through two distinct pathways. One is induced by 53BP1, that remodels the stalled RF without inducing DNA breakage, and the second is mediated by BRCA1, that triggers the fork-cleavage-coupled break-induced replication (BIR) pathway, mediated by the endonuclease MUS81 (61). In the early stage of replication stress, the balance favors the 53BP1-dependent pathway, but when replication stress is prolonged, PLK1 determines the switch from 53BP1-mediated pathway to the BRCA1-cleavage pathway (61).

These findings are consistent with PLK1 regulatory function not only in DDR through the HR pathway, but also in the replication stress response when replication origins stall in the presence of a DSB. In the metazoan, the ATM/ATR-dependent intra-S-phase checkpoint usually inhibits the firing of new replication origins, but in the presence of replication stress the dormant origins can be activated, following transient suppression of the intra-S-phase checkpoint, in order to preserve genomic stability (62). ATM/ATR phosphorylate MCM2, promoting PLK1 binding to the MCM complex (63, 64). PLK1 and the MCM complex, localized at the stalled RFs, promote the release of CHK1-mediated suppression of nearby dormant origins, even if this later interaction is not completely explained. PLK1-mediated phosphorylation of RAD51 is important for the protection of nascent ssDNA at stalled RFs following hydroxyurea (HU) treatment, in a BRCA2-dependent manner, from late-S-phase to mitosis, to improve genomic stability (65). All this evidence supports the critical role of PLK1 in DDR and consequently in maintaining genomic stability.

## Other Functions of Plk1

### PLK1 and Epithelial-to-Mesenchymal Transition

EMT is a process by which epithelial cells lose their characteristics (e.g. cell-cell and cell-extracellular matrix adhesion, cell polarity and morphology) and acquire a mesenchymal cell phenotype (fibroblast-like morphology, increased cell-matrix adhesions, and motility). Although EMT is involved in fundamental early processes including embryonic development, tissue formation and tissue fibrosis, it has also be implicated in tumor cell growth and proliferation, drug resistance and metastasis formation (66–68). In the last years, PLK1 emerged as one of the triggers of this process (69) (**Figure 2**).

**Figure 2:** Main PLK1 functions in cellular processes beyond mitosis and DNA damage response. PLK1 interacts with several intracellular factors regulating cell death pathways (i.e. apoptosis, autophagy and pyroptosis), immune response, inflammation and epithelial to mesenchymal transition.

The molecular evidence of EMT is downregulation of epithelial markers, such as E-cadherin and some cytokeratin isoforms, and the overexpression of mesenchymal markers, such as N-cadherin and vimentin (70). PLK1 overexpression in prostate epithelial cells was associated with downregulation of E-cadherin and cytokeratin 19 and upregulation of N-cadherin, vimentin, fibronectin, and SM22, while its downregulation enhanced epithelial characteristics, reversed the EMT and inhibited cell motility (71). A comparison between cells expressing constitutively active wild-type or kinase-defective protein indicated that the induction of EMT requires PLK1-mediated phosphorylation events. In particular, PLK1 phosphorylates cRAF, which induces the MEK/ERK cascade eventually activating ZEB1 and ZEB2 transcription factors, leading to the expression of EMT genes (71).

The PLK1-driven EMT has also been reported in gastric carcinoma cells, where the overexpression of PLK1 induced down-regulation of E-cadherin and up-regulation of N-cadherin, Slug and Twist, through the induction of PLK1-mediated AKT phosphorylation (72). Instead, in non-small cell lung cancer (NSCLC) the role of PLK1 in promoting EMT and metastasis formation correlated with upregulation of the TGFβ/SMAD pathway (73, 74). Shin et al. demonstrated that the active PLK1 (p-Thr210 PLK1) is abundant in TGFβ-induced metastatic NSCLC and its presence promoted *in vivo* metastasis formation; active PLK1 led to an increase of the levels of TGFβ cascade effectors, including SNAI1, SNAI2, ZEB1, CDH2, IL11, and TNFAIP6, whose depletion resulted in a reversion of the EMT induced by active PLK1 (73). Moreover, PLK1 is responsible of the phosphorylation of FoxM1 (31), another promoter of EMT in different tumor types including lung (75, 76), prostate (77), gastrointestinal cancer (78), pancreas (79), glioblastoma (80) and glioma (81). Taken together, PLK1 activity promotes the epithelial-mesenchymal transition in different type of tumors.

### PLK1 and Cell Death Pathways

Cell death through regulated molecular pathways (i.e. autophagy and apoptosis) occurs in physiological conditions in order to preserve the organism’s homeostasis. However, in cancer cells these pathways are impaired, especially after drug treatment (82, 83).

PLK1 has a role of in the inhibition of cell death pathways including autophagy and apoptosis (**Figure 2**). Autophagy is a conserved, adaptive process of self-degradation for the maintenance of cellular homeostasis, that can also occur in response to cellular stress (i.e. nutrient deprivation, growth factor depletion, infection, hypoxia) (84). Alterations in this pathway can lead to the initiation and development of tumors. Among the signaling pathways involved in this process, the mTOR (mammalian target of rapamycin) pathway is the most important and conserved. The Ser/Thr kinase mTOR and its regulatory protein RAPTOR forms the multiprotein complex mTORC1, which can inhibit autophagy under normal conditions (85). In HeLa cells PLK1 was identified as a physical interactor of mTORC1 by mTOR direct binding (86). In that study, Ruf et al. demonstrated that PLK1 and mTORC1 co-localize in the lysosomes and that the inhibition of PLK1 by shRNA or drug treatment promoted mTOR lysosomal localization and reduced autophagy, while PLK1 overexpression inhibited mTORC1 and contributed positively to autophagy.

In glioma cells, knock-out of PLK1 by shRNA had an inhibitory effect on autophagy through phosphorylation of the mTORC1 substrate RPS6KB (87). On the other hand, in esophageal squamous cell carcinoma (ESCC) (88) and acute myeloid leukemia (AML) cells (89) there was an opposite correlation between mTOR and PLK1 in autophagy. In ESCC, the suppression of PLK1 downregulated mTOR activity, suggesting that PLK1 activates the mTOR signaling pathway both *in vitro* and *in vivo*. Similarly, in AML cells, the inhibition of PLK1 led to autophagy induction through mTORC1 dephosphorylation.

In a recent study by Wang et al. PLK1 inhibition suppressed radiation-induced autophagy in breast cancer cells, while its overexpression increased it (90). In osteosarcoma cells, PLK1 overexpression led to downregulation of autophagy-related proteins such as Beclin-1 and LC3-II (91) by regulating MYC stabilization (92). Similarly, in ovarian clear cells carcinoma, PLK1 silencing resulted in lower LC3B-II induction with an impairment of autophagy (93). In that study, PLK1 knock-down correlated with an increase of apoptotic cells due to an increase of caspase 3 cleavage. These contrasting evidence may suggest that the PLK1-mediated regulation of autophagy may be cell type-specific, but further investigations are still needed.

Apoptosis is a programmed cell death pathway that leads to orderly and efficient removal of damaged cells, such as those following DNA damage or during development (94). The apoptosis machinery is complex and involves many signaling pathways, whose alterations result in deregulation of development, progression of cancer, and tumor resistance to therapy, and has been listed as an hallmark of cancer (95).

The tumor-suppressor p53 mediates apoptosis by activating mitochondrial and death receptor-induced apoptotic pathways with the activation of caspase signaling (96). Ando et al. not only demonstrated the physical interaction between PLK1 and p53, but also showed that the pro-apoptotic function of p53 was inhibited by the kinase activity of PLK1 (97). In castration-resistant prostate cancer cells the inhibition of PLK1 by the small molecule BI2536 resulted in an increased p53-induced cellular death (98). Recently, in TNBC too, the downregulation of PLK1 by the microRNA miR-183-5p resulted in an increase of apoptosis through the DNMT1-p53 axis (99).

As a member of the p53 family, p73 as well can induce apoptosis (100). PLK1 inhibits p73 pro-apoptotic activity by phosphorylating at Thr27 (101), while its silencing through small interference RNA led to increased p73 levels (102).

PLK1 seems also to interfere with caspase activity. During mitosis cyclinB1/CDK1 complex phosphorylates the pro-caspase-8, generating a phospho-epitope for the binding of PLK1, that interferes with caspase-8 auto-activation resulting in inhibition of apoptosis (103). In human airway smooth muscle cells the expression of PLK1 correlated with increased levels of pro-caspase-9 and -3, as indicated by the enhanced apoptosis resulting from PLK1 knockdown (104).

A regulatory role of PLK1 in cell death has also been described through action on other interactors. In renal carcinoma cells PLK1 suppressed apoptosis by phosphorylating the mini-chromosome maintenance 3 protein (MCM3) (105), while in lung adenocarcinoma it regulated the expression of karyopherin beta 1 (KPNB1) (106). However, in contrast with previous evidence, in some other studies PLK1 seemed to promote cell death. It was reported that PLK1 phosphorylates the Fas-associated death domain (FADD) after treatment with taxol, triggering caspase-mediated cell death (107, 108). In HeLa cells, phosphorylated FADD induces not only caspase-8, but also causes proteasomal degradation of PLK1 as a negative feedback loop (107). Similarly, Gupta et al. demonstrated that PLK1 modulates the phosphorylation of the receptor-interacting protein kinase 3 (RIPK3) involved in the induction of different cell death pathways (109).

Beside apoptosis, pyroptosis (or inflammatory cell necrosis) is another programmed cell death pathway activated by the inflammatory caspases (caspase-1 and caspase-11 in mice and caspase-1, caspase-4, and caspase-5 in humans) (110). Activation of this pathway causes cells to start swell, with a rapid destabilization of plasma membrane integrity, leading to the release of cell content including danger-associated molecular patterns (DAMPs) and cytokines that trigger a robust inflammatory response (111). Pyroptosis can also influence the proliferation, invasion and metastasis of different tumors, as recently reviewed (112). Inhibition of PLK1 by BI2536 treatment in esophageal squamous cell carcinoma (ESCC) induced pyroptosis both *in vitro* and *in vivo* through the BAX/caspase-3/GSDME pathway and boosted the sensitivity to cisplatin (113).

### PLK1 and Immune Response/Inflammatory Signaling

In recent years, the immune response has emerged as an important factor in tumor progression and treatment (114, 115). The possible role of PLK1 in modulating immunity has also been investigated.

From a screening in more than 30 different cancers, a correlation was seen between high levels of PLK1 and inhibition of immune cell infiltration and antitumor immunity (116). In particular, tumors with elevated expression of PLK1 displayed lower immune activity, such as lower expression of Human Leukocyte Antigens (HLA), fewer B cells, NK cells and tumor-infiltrating lymphocytes and reduction of T-regulatory cells. In addition, *in vitro* treatment with PLK1 inhibitors upregulated the expression of HLA molecules in different cancer cells. In lung cancer PLK1 expression not only negatively correlated with numerous immune cell lineages, but was also crucial in antigen processing and presentation (117). Its inhibition with BI2536 resulted in increased maturation of dendritic cells (DC) and enrichment of T cells infiltration, and promoted immune cell infiltration and activation *in vivo*, supporting the possibility that PLK1 blockade may act as an immune activator. In hepatocellular carcinoma the PLK1/PTEN axis activated by the cell transformation sequence 2 (ECT2) protein promoted M2 macrophage polarization, resulting in suppression of both NK and T cells functions (118).

The nuclear factor kappa light chain enhancer of activated B cells (NF-κB) is an ubiquitous transcription factor known for its role in the regulation of inflammation and innate immunity, since its stimulation triggers the expression of inflammatory mediators including cytokines, chemokines and cell adhesion molecules (119). The activity of NF-κB is tightly regulated through inhibitory IκB proteins and the kinase that phosphorylates IκBs, namely, the IκB kinase (IKK) complex. Stimulation through TLR4, TNF-α receptor (TNFR) and interleukin-1 receptor (IL-1R) activation leads to phosphorylation of IKK and release of NF-κB dimers (119).

In the last few years, PLK1 has been reported as a negative regulator of NF-κB transcriptional activation. Constitutively active expression of PLK1 in mammalian cells reduced tumor necrosis factor (TNF)-induced IKK activation, through inhibition of cyclin D1 expression, resulting in decreased phosphorylation of endogenous IκBα, and consequently reduced NF-κB activation (120). However, the suppression by PLK1 on the NF-κB signaling pathway was also promoted by the interaction of PLK1 with the TRAF-associated NF-κB activator (TANK) (121). Mechanistically, PLK1 binds the IKK adaptor protein NEMO, preventing its ubiquitination through the formation of a ternary complex with TANK, negatively regulating the TNF-induced IKK activation.

PLK1 also regulates the NF-κВ and the interferon regulatory factor 3 (IRF3) pathway by modulating mitochondrial antiviral-signaling (MAVS) protein activity (122). Briefly, the PBD domain of PLK1 associates with two different domains of MAVS in both dependent and independent phosphorylation events. The phospho-independent binding strongly disrupts the association of MAVS with its downstream partner TRAF3, which is essential for activation of an alternative IKK complex responsible for IRF3 phosphorylation. In **Figure 2** are graphically summarized the interactions of PLK1 with factors involved in the immune response and NF-κB activator pathway.

## PLK1 Inhibitors

Considering the pleiotropic roles of PLK1 in many cellular pathways whose involvement in cancer has been clearly demonstrated, PLK1 is a potential therapeutic target and in the last decade various PLK1 inhibitors have been developed by drug companies and academic research groups.

Two types of small molecule have been developed as PLK1 inhibitors: ATP-competitors target the kinase domain of the protein and non-ATP competitors target the PBD domain. Several drugs targeting the ATP-binding domain have been identified and some have progressed to clinical trials. However, there are important potential drawbacks with these molecules as they also inhibit the catalytic domain of the other PLKs; this could increase the toxic side effects and, in some cases-considering the different possible contrasting effects of the PLKs- might reduce the antitumor effects. In addition, like with other ATP competitors, point mutation (C67V) in the ATP-binding domain can confer resistance to other structurally unrelated ATP-inhibitors (123). Inhibitors targeting the PBD domain need to be more specific, as the PLK1-3 PBDs have unique substrate specificity allowing the design of target therapeutics (124), and could potentially suggest a novel biological basis on the molecular recognition of PLK1 and its substrates.

Different compounds have been synthesized (6, 125, 126). At the moment there are more than ten available PLK1 specific inhibitors, four of which (BI2536, BI6727-volasertib, GSK461364 and NMS-1286937-onvasertib- all ATP competitors) have reached the clinical trials (listed in **Table 1**).

**Table 1:** Clinical trials based on PLK1 inhibitors.

NCT number	Phase	Disease	PLK1i	Ref
NCT02211859	I	Advanced solid tumors	BI2536	(127)
NCT02211872	I	Advanced solid tumors	BI2536	(128)
NCT00412880	II	Small cell lung cancer	BI2536	(129)
NCT01662505	I	Acute myeloid leukaemia	BI6727 (Volasertib)	(130)
NCT00804856	I/IIa	Acute myeloid leukaemia	BI6727 (Volasertib)	(131)
NCT01023958	II	Urothelial cancer	BI6727 (Volasertib)	(132)
NCT00824408	II	NSCLC	BI6727 (Volasertib)	(133)
NCT01014429	I	Advanced solid tumors	NMS-1286937 (Onvansertib)	(134)
NCT00536835	I	Advanced solid tumors	GSK461364	(135)
NCT01179399	I	Advanced solid tumors	TAK960	Not yet published
NCT01538537	I	Advanced solid tumors	ON01910 (Rigosertib)	(136, 137)
NCT00854646	I/II	Myelodysplastic syndrome Acute myeloid leukemia	ON01910 (Rigosertib)	(138)
NCT01168011	I	Advanced solid tumors	ON01910 (Rigosertib)	(139)

BI2536 is an adenosine triphosphate (ATP)–competitive kinase inhibitor derived from the novel chemical series of dihydropteridinone (140). It is a potent PLK1 inhibitor. BI2536 induces G2/M arrest and the formation of abnormal mitotic figures, such as monopolar spindles (141). Its effect has been observed *in vitro*, at nanomolar concentrations, and also *in vivo* (at a nanomolar concentration as well) with an acceptable safety profile (140). In Phase I studies, BI2536’s dose-limiting toxicity was reversible neutropenia, the most frequent adverse event at the maximum tolerated dose (grade 3 to 4; 56%); nausea, fatigue and anorexia were also frequent, but mostly mild to moderate (127). The toxicity profile was similar when combined with pemetrexed in NSCLC patients (142). These studies hinted at antitumor activities. However, in 21 patients with relapsed small-cell lung cancer enrolled in a Phase II study with BI2536, no responses were observed and disease progressed in all the patients (129).

No objective response or considerable tumor regression was observed in patients with advanced solid tumors (colorectal, melanoma, hepatoma and ovarian cancer) in a Phase I study (128). There was also no activity in chemo-naïve patients with unresectable exocrine adenocarcinoma of the pancreas (6). All these data were discouraging and have not fostered any further drug clinical investigation.

Volasertib (BI6727) is an ATP-competitive kinase inhibitor belonging to the same dihydropteridinone class as BI2536 (143), whose development was discontinued in favor of volasertib. Volasertib cytotoxic effects have been observed at nanomolar concentrations (144) in acute myeloid leukemia cells (144), and in carcinoma cancer cells (145) with both the induction of cell cycle arrest and cell death (146).

Volasertib had a better pharmacokinetic profile than BI2536, with a high volume of distribution, deep tissue penetration, and a long terminal half-life (147). *In vivo* preclinical data indicated that volasertib has antitumor activities in different tumors with quite a safe toxicological profile (148), fostering its clinical development. Phase I studies in monotherapy defined the maximum tolerated doses (400-450 mg every two or three weeks), with the most frequent side effects being haematological toxicities (anemia, neutropenia, thrombocytopenia), being reversible and manageable with standard care (130, 131). Phase II studies as single agent, however, showed only modest antitumor activity (132, 133).

NMS-1286937 (onvansertib), a pyrazoloquinazoline, is a third generation PLK1 ATP-competitor with an *in vitro* IC50 of 36 nmol/L, and had a strong cytotoxic effect in AML cells, for which it was originally registered by FDA as orphan drug (149). Onvansertib induced a mitotic cell-cycle arrest followed by apoptosis in cancer cells; it inhibited xenograft tumor growth at well tolerated oral doses (150). In addition, it potentiated cytarabine antitumor activity in a disseminated model of AML (149). On the basis of these promising results a Phase I trial with escalating drug doses was conducted in 21 patients with advanced tumors (134). This allowed the definition of the maximum tolerated dose, and dose limiting toxicities (mainly thrombocytopenia and neutropenia) with disease stabilization in several patients as the best treatment response (134).

GSK461364 is thiophene amide, an ATP-competitor PLK1 inhibitor, which promotes G2/M arrest in tumor tissues (151); in addition, the drug enhanced the radio sensitivity of breast cancer cells *in vivo* (90). A Phase I trial was conducted with two different schedules and GSK461364 doses in 40 patients with solid tumors; the dose-limiting toxicities were haematological (neutropenia and trombocytopenia) and venous thrombotic emboli; prolonged disease stabilization was the best activity reported in 15% of patients, including four with esophageal cancers (135).

Tak960 is a recently synthesized ATP-competitor PLK1 inhibitor, orally available and PLK1 selective (152). Tak960 arrests the cell cycle in G2/M phase, and accumulates cells with aberrant spindles (153). It has been shown *in vitro* cytototoxic activity in different cells and xenograft models, with favourable tolerability and PK/PD profiles (153). It is currently under Phase I investigation in advanced non-haematological malignancies (NCT01179399).

Rigosertib (ON01910) is a benzyl sulfone analog that acts as a Ras mimetic, and non- ATP- competitive molecule inhibiting both PLK1 and PI3K (154). Rigosertib induces mitotic arrest in different cancer cells by inducing spindle abnormalities, cell cycle arrest and apoptosis (155–157).

In Phase I/II trials was well tolerated and showed some activity in selected patients with advanced solid tumors (136, 137). Rigosertib had good tolerance in high-risk myelodysplastic syndrome and AML, with hints of antitumor activity (138). The most common side effect was urinary toxicity (139). In a Phase I trial, rigosertib’s most common side effects involved urothelial irritation and the dose-limiting toxicities were haematuria and dysuria (139).

Inhibition of the PBD domain of PLK1 is another strategy to target PLK1. As said, this domain is a docking site for phosphorylated substrates and is a druggable interface, as demonstrated in different studies (139, 154, 158). Poloxin, a synthetic thymoquinone derivative, was one of the first compounds shown to interfere with the interaction between the PBD of PLK1 and an optimal phosphor-peptide (126). It was later seen that also thymoquinone, with its similar chemical structure, had similar effects. Poloxin caused centrosome fragmentation, abnormal spindle, chromosome misalignment, mitotic arrest, and apoptosis in cancer cell lines and had a significantly effect in suppressing xenograft growth *in vivo* (159).

Different inhibitors of PLK1 have been generated through high-throughput screening approaches (9, 126, 155). However, many of these molecules could not be further developed because they had only modest activity in preclinical models and were shown to be non-specific protein alkylators (160). Recently, using REPLACE (Replacement with Partial Ligand Alternatives through Computational Enrichment), PLK1 inhibitors have been synthesized and showed to have promising PBD binding activity and cytotoxic activity in *in vitro* cell lines (6).

## PLK1 Inhibition Combination Therapies

The use of PLK1 inhibitors has been widely used in preclinical studies, but has not been successfully translated to the clinic on account of its limited effect and resistance [reviewed in (161)]. To overcome this, researchers have started to investigate the possibility of combining PLK1 inhibitors with other agents. Combination therapy offers the opportunity to target different pathways, to eliminate different cancer cell populations, and possibly obtain additive/synergistic anticancer effects.

Investigations have also been examined possibility to boosting the response to therapy in different cancers by combining PLK1 inhibitors with chemotherapies (**Table 2**). The most widely studied PLK1 inhibitors were BI2536, volasertib and onvansertib. The ability of PLK1 inhibitors to induce G2/M cell cycle arrest was exploited in cisplatin-resistant gastric cancer cells, where the combination of BI2536 and cisplatin inhibited cell growth and invasion ability (162). Volasertib too potentiated the activity of cisplatin in cervical cancer (167).

**Table 2:** Combination strategies with PLK1 inhibitors: *in vitro* data.

PLK1 inhibitor	Agent	Disease	Ref
volasertib/BI6727	cisplatin	gastric cancer	(162)
	doxorubicine	triple negative breast cancer	(163)
	cyclophosphamide	triple negative breast cancer	(163)
	fadusil (ROCK inhibitor)	lung cancer	(164)
	olaparib	castration-resistant prostate cancer	(165)
	eribulin	rabdomyosarcoma	(166)
	cisplatin	cervical cancer	(167)
	paclitaxel	ovarian cancer	(168)
	JTP-74017 (MEK inhibitor)	NRAS mutant melanoma	(169)
	MK0752 (NOTCH inhibitor)	melanoma	(170)
	erlotinib	NSCLC	(171)
	P22077 (USP inhibitor)	lung cancer	(172)
onvansertib/NMS-1286937	paclitaxel	triple negative breast cancer	(173)
	docetaxel	triple negative breast cancer	(173)
GSK461364	paclitaxel	triple negative breast cancer	(173)
	docetaxel	triple negative breast cancer	(173)
	BRD4 inhibitor	castration-resistant prostate cancer	(174)

In ovarian cancer cells with CCNE1 amplification the combination of volasertib with paclitaxel synergistically triggered mitotic arrest, initiating mitochondrial apoptosis (168). Onvansertib too showed synergistic activity with paclitaxel, as reported by different groups, including ours (173, 175). Giordano et al. tested onvansertib and another PLK1 inhibitor (GSK461364) in combination with taxanes (paclitaxel and docetaxel) in a set of triple negative breast cancer cell lines *in vitro* and *in vivo*. Both the PLK1 inhibitors synergized with taxanes specifically inhibiting the G2/M transition, inducing aberrant mitotic exit and apoptosis, and also eliminating stem-like resistant clones (173). In another work, our group further showed that onvansertib and paclitaxel acted synergistically both *in vitro* and *in vivo* in xenografts, causing tumor regression and tumor growth inhibition in a model of mucinous ovarian cancer (175). The PLK1 inhibitor GSK461364 was also tested in combination with a BRD4 small inhibitor in castration-resistant prostate cancer both *in vitro* and *in vivo*, showing a strong synergistic effect (174).

Dual targeting of mitosis caused a synergistic induction of apoptosis for BI2536-eribulin co-treatment in rhabdomyosarcoma *in vitro* (166). In a triple negative breast cancer, the PLK1 inhibitor BI2536 impaired tumor growth also *in vivo* as single agent, but when combined with doxorubicin and cyclophosphamide this treatment gave a faster complete response and prevented relapses (163).

The possibility of combining PLK1 inhibitors to increase its efficacy and avoid the development of resistance was also tested in combination with targeted therapies. BI2536 was combined in tumors with defined pathways alterations (i.e. *KRAS* mutated cancers). Wang et al. showed that the inhibition of PLK1 and ROCK in *KRAS*-mutated lung cancer cells (but not in the wild type), through the upregulation of p21 protein, reduced viability (164). BI2536 was also tested with olaparib, a FDA-approved PARP inhibitor, mostly used in BRCA-deficient tumors and this combination synergistically inhibited the growth of xenograft tumors derived from *BRCA*-mutated castration-resistant prostate cancer (165).

In *NRAS* mutant melanoma the combination of volasertib and a MEK inhibitor (JTP-74017) had antitumor effects both *in vitro* and *in vivo* (169). Again, the synergistic effect was due to cell cycle arrest and greater induction of apoptosis. Su et al. found that the expression of PLK1 and NOTCH was associated with poor overall and disease-free survival in melanoma, and the combination of BI6727 with the NOTCH inhibitor MK0752 resulted in a synergistic antiproliferative response in *BRAF* mutated, *BRAF* and *TP53* mutated, and *NRAS* mutated melanoma cells (170).

In different NSCLC cells mutated in the epidermal growth factor receptor (EGFR) volasertib reversed resistance to erlotinib, causing G2/M arrest and apoptosis, and reduced tumor growth *in vivo* (171). Volasertib had a strong synergistic effect also when combined with a USP7 inhibitor, counteracting resistance to taxane. In paclitaxel resistant lung cancer cells the combination counteracted the resistance to mitotic catastrophe through downregulation of MDR1/ABCB1 protein (172).

All these preclinical studies uphold the use of PLK1 inhibitor combinations in clinic (**Table 3**). In a Phase I trial BI6727 was combined with escalating doses of decitabine to investigate the maximum tolerated dose, safety and pharmacokinetics (176). The drug was also tested in a Phase II trial in AML in combination with low-dose cytarabine (177). Patients treated with the combination had a higher response rate (31%) than with low-dose cytarabine monotherapy (13%). This study launched a Phase III trial (NCT01721876), which aimed to investigate the efficacy, safety, and pharmacokinetics of volasertib with low-dose cytarabine in patients over 65 years of age with untreated AML (178). In 2013 the Food and Drug Administration granted volasertib breakthrough therapy status for combined treatment with cytarabine in AML.

**Table 3:** Clinical trials based on PLK1 inhibition combination therapy.

NCT number	Phase	Disease	PLK1i	Other therapy	Ref
NCT02003573	I	acute myeloid leukemia	volasertib	escalating doses of decitabine	(176)
NCT00804856	II	acute myeloid leukemia	volasertib	LDAC*	(177)
NCT01721876	III	acute myeloid leukemia	volasertib	LDAC	(178)
NCT03303339	I	acute myeloid leukemia	onvansertib	LDAC/decitabine	(179)
NCT00824408	I	NSCLC	volasertib	pemetrexed	(133)
NCT01206816	I	solid advanced tumors	volasertib	afatinib	(180)
NCT01022853	I	advanced metastatic solid tumors	volasertib	nintedanib	(181)
NCT01772563	I	advanced metastatic solid tumors	volasertib	itraconazole	(182)

*low dose cytarabine

Escalating doses of the third-generation PLK1 inhibitor onvansertib were tested in a Phase Ib study, alone and in combination with low-dose cytarabine (LDAC) or decitabine for AML. The combination was well tolerated and achieved a 24% complete remission rate (5 of the 21 evaluable patients) (179), supporting its further investigation in the ongoing phase II trial. Recently onvansertib was granted by a Fast Track Designation for the second-line treatment of patients with *KRAS*-mutant metastatic colorectal cancer in combination with 5-fluorouracil, leucovorin, irinotecan and bevacizumab (183).

The combination of PLK1 inhibitors with other drugs was also studied in solid tumors, but so far, they have not gone beyond Phase I. The combination of volasertib with pemetrexed for advanced/metastatic NSCLC did not have any greater toxicity, but did not improve the efficacy compared with pemetrexed single-agent (133). A combination of volasertib and afatinib (an oral ERBB family blocker) was tested in a Phase I trial in 57 patients with advanced solid tumors. However, only two patients achieved partial responses and eight experienced stable disease (180). Volasertib was recently combined with nintedanib a potent inhibitor of PDGF, VEGF and bFGF receptor, in patients with advanced solid tumors in a Phase I dose escalation study. It gave a well-tolerated safety profile with no unexpected or overlapping side effects and with significant tumor stabilization (181).

## Concluding Remarks

PLK1 is the most studied of the PLKs. Its main role is in the progression of mitosis, with an established regulatory function in mitotic entry, maturation of the centrosome, spindle assembly and cytokinesis. Recent works implicate PLK1 in many of the cellular pathways as we have discussed briefly. While PLK1 mutations are extremely rare in human cancers, it is often found overexpressed, especially in advanced cancers. This overexpression is often correlated with aggressiveness and poor patient prognosis. These evidence all have points to PLK1 as a promising therapeutic target in oncology. Small interfering RNA, CRISPR/Cas9 deleted PLK1 and chemical inhibitors of PLK1 have an impact on cell proliferation, cause mitotic arrest, cell death and *in vivo* tumor growth inhibition.

As summarized here, a number of inhibitors (ATP-competitors) have been synthesized and showed activity in both *in vitro* and *in vivo* preclinical models, fostering their clinical development. Their toxicological profiles are quite similar, the most frequent reported dose limiting toxicities in most cases being haematological toxicities (neutropenia and thrombocytopenia). As regards clinical efficacy, the results were not as expected when used in second and higher lines of therapy. However, there were hints of activity in specific subsets of patients and this has allowed volasertib and onvansertib to be granted by FDA as respectively breakthrough therapy and orphan drug status. The various new functions of PLK1 in many different cellular pathways suggest potential new combination approaches aimed at target tumor cell vulnerabilities/hallmarks (for example, with immunotherapy).

Lastly, the search for PLK1 synthetic lethal partners could be another strategy, still little developed. Recent data suggest this could be a complementary, efficacious approach. An unforeseen synthetic lethal interaction has in fact been reported between PLK1 and BRCA1 from screening a kinase inhibitors library (184). The authors found that BRCA1 downregulation and inhibition of PLK1 induced aberrant mitotic phenotypes, centrosomal duplication and altered cytokinesis, resulting in reduced clonogenicity of these cells. These data suggest the use of PLK1 inhibitors in subsets of patients (*BRCA1*-mutated, in triple negative breast and ovarian cancer). Emerging evidence also suggest that tumors with activated KRAS seem to be addicted to PLK1 activity (185) potentially opening the way to target KRAS mutated tumors with PLK1 inhibitors.

## Author Contributions

MC, SP, GD, FG, FR and MB contributed conception and design of the review; MC, SP, GD, FG and FR wrote the manuscript. All authors contributed to manuscript revision, read and approved the submitted version.

## Funding

We acknowledge the support by the Italian Association for Cancer Research (AIRC, IG19797 project, PI GD; AIRC, IG24347, PI MB).

## Conflict of Interest

The authors declare that the research was conducted in the absence of any commercial or financial relationships that could be construed as a potential conflict of interest.

## Publisher’s Note

All claims expressed in this article are solely those of the authors and do not necessarily represent those of their affiliated organizations, or those of the publisher, the editors and the reviewers. Any product that may be evaluated in this article, or claim that may be made by its manufacturer, is not guaranteed or endorsed by the publisher.
